RETRACTED

# Changes in Thrombelastography in Patients with Acute Exacerbation of Chronic Obstructive Pulmonary Disease and the Relationship with Lung Function

**DOI:** 10.1155/2022/4313394

**Published:** 2022-11-10

**Authors:** Yan Zhou, Jing Yu, Haiying Zhou

**Affiliations:** Department of Respiratory and Critical Care Medicine, Zhuji People's Hospital, Zhuji, Zhejiang Province 311800, China

## Abstract

**Purpose:**

To analyze the changes in thrombelastography (TEG) in patients with acute exacerbation of chronic obstructive pulmonary disease (AECOPD) and the relationship with indicators related to lung function.

**Methods:**

100 patients with AECOPD admitted to our hospital from May 2021 to May 2022 were selected as the AE group, and another 80 patients with a stable phase of COPD in the same period were selected as the SP group. Fresh blood specimens were collected from both groups, and TEG-related indicators (*R* value, *K* value, *α*-angle, MA value) were measured using the TEG technique, and lung function-related indicators (FEV1, FVC, FEV1/FVC, FEV1%) were measured using a lung function meter, and the correlation between TEG-related indicators and lung function-related indicators was analyzed.

**Results:**

Patients in the AE group had lower *R* and *K* values and higher *α*-angle and MA values than those in the SP group, all with statistically significant differences (*P* < 0.05). Patients in the AE group had lower FEV1, FVC, FEV1/FVC, and FEV1% levels than those in the SP group, all with statistically significant differences (*P* < 0.05). Correlation analysis showed that the *R* value in TEG of AECOPD patients was positively correlated with pulmonary function-related indicators (FEV1, FVC, FEV1/FVC, FEV1%) (*r* = 0.565, 0.529, 0.447, 0.527, all *P* < 0.001); *K* value was positively correlated with pulmonary function-related indicators (FEV1, FVC, FEV1/FVC, FEV1%) (*r* = 0.512, 0.567, 0.459, 0.439, all *P* < 0.001); *α*-angle was inversely correlated with pulmonary function-related indicators (FEV1, FVC, FEV1/FVC, FEV1%) (*r* = −0.498, −0.372, −0.408, −0.424, all *P* < 0.001); MA value was inversely correlated with lung function-related indicators (FEV1, FVC, FEV1/FVC, FEV1%) (*r* = −0.459, −0.429, −0.394, −0.403, all *P* < 0.001).

**Conclusion:**

There is a correlation between TEG-related indicators and lung function-related indicators in AECOPD patients, both of which can guide the diagnosis and treatment process of the disease and are worthy of clinical promotion. The clinical registration number is EA2021086.

## 1. Introduction

Chronic obstructive pulmonary disease (COPD) is a common, preventable, and treatable respiratory disease characterized by persistent respiratory symptoms and airflow limitation and is a global public health challenge due to its high prevalence, disability, and mortality. Cross-sectional foreign epidemiological studies have shown that the prevalence of COPD is 3.6% in adults aged 45 years and older and increases with age [1]. In China, approximately 100 million people suffer from COPD, with an overall prevalence of 8.6% [2]. And by 2020, COPD becomes the third most deadly disease in the world [3]. In the course of COPD, patients sometimes have aggravated respiratory symptoms and progressive decline in lung function, and even causes respiratory failure and systemic inflammatory response syndrome, which is called acute exacerbation of chronic obstructive pulmonary disease (AECOPD) [4, 5]. At present, AECOPD can be diagnosed and evaluated clinically by serum inflammatory factor levels and lung function indicators [6, 7]. However, with the complex causes of acute exacerbations in COPD patients, the lack of specificity of inflammatory factors and the physical requirements of pulmonary function tests for patients, there is a clinical need to find more specific and sensitive indicators to support diagnosis and assessment. Previous studies [8] have pointed out that patients with COPD have abnormal coagulation-fibrinolysis function, and the high coagulation state in the acute exacerbation period may lead to pulmonary hypertension, right heart injury, pulmonary vascular microthrombotic embolism, etc., which may affect the prognosis of patients. It is therefore essential to assess the coagulation status of patients with AECOPD. However, changes in the four coagulation indicators only reflect a certain stage of the coagulation mechanism and do not reflect the coagulation status within the blood cells, which is a limitation. Thrombelastography (TEG) is an immediate bedside test, which uses whole blood specimens for testing and includes the influence of blood cells as well as plasma components on the coagulation process, simulating the entire process in the human body from the beginning of coagulation to fibrinolysis and can effectively reflect the function of coagulation factors, fibrinogen, platelets, etc., making up for the deficiencies of the four indicators of coagulation [9, 10]. This study analyses the changes in TEG and the relationship with lung function-related indicators in patients with AECOPD and evaluates the value of TEG in this group of patients. It is reported as follows:

RETRACTED

## 2. Materials and Methods

### 2.1. Research Object

100 patients with AECOPD admitted to our hospital from May 2021 to May 2022 were selected as the AE group, and another 80 patients with a stable phase of COPD in the same period were selected as the SP group. Inclusion criteria were as follows: (1) diagnostic criteria for AECOPD referred to the 2018 edition of the global initiative for chronic obstructive lung disease (GOLD) [11]: patients with progressively worsening dyspnea, chronic cough or sputum; history of long-term smoking and occupational or environmental exposure to noxious gases; pulmonary function tests showing FEV1/FVC < 0.70 after inhalation of bronchodilators, excluding other diseases causing airflow limitation; (2) those with complete information on TEG, pulmonary function tests, coagulation tests, and arterial blood gas analysis; (3) those who voluntarily participated in this study. Exclusion criteria were as follows: (1) combination of other acute events such as acute stroke and acute myocardial infarction; (2) combination of bronchiectasis, bronchial asthma, and active tuberculosis; (3) previous history of venous thromboembolism, cerebral infarction, myocardial infarction, etc.; (4) those who had taken antiplatelet agents or anticoagulants within the last 2 weeks; (5) history of major surgical trauma within 6 months; (6) combination of tumor and immune system; (7) those with significant hematological disorders or severe hepatic or renal insufficiency.

### 2.2. Research Methods

#### 2.2.1. Baseline Information Collection

Baseline information on gender, age, body mass index (BMI = kg/m^2^), duration of illness, number of days of exacerbation, and smoking history were collected from all patients. The comparison of baseline information between the two groups is shown in Table 1 and was not statistically significant (*P* > 0.05) and was comparable.

#### 2.2.2. TEG Examination

Fresh blood specimens were collected from both groups in the early morning of the day following enrollment, and TEG-related indicators, including reaction of blood coagulation time (*R* value), kinetics time (*K* value), alpha coagulation angle (*α*-angle), and maximum amplitude (MA value), were measured using a TEG 5000 thromboelastography. The normal reference ranges for each of the TEG indicators and the significance of their detection are shown in Table 2.

#### 2.2.3. Pulmonary Function Examination

In the awake state of all patients, lung function-related indicators were measured using the German JAEGFR lung function test, including forced expiratory volume in one second (FEV1), forced vital capacity (FVC), FEV1/FVC, and FEV1 as a percentage of the expected value (FEV1%).

### 2.3. Statistical Methods

SPSS 22.0 was applied to analyze the statistical data and GraphPad Prism 8.0.2.263 was applied to plot the graphs. The count data in the baseline information was expressed in (%), using the *χ*^2^ test. The measurement data was expressed in ($\bar{x}$±*s*) and tested with *t*. The correlation between TEG-related indicators and lung function-related indicators was analyzed by Pearson correlation. *P* < 0.05 was statistically significant.

RETRACTED

## 3. Results

### 3.1. Comparison of TEG Parameters for Both Groups

Patients in the AE group had lower *R* and *K* values and higher *α*-angle and MA values than those in the SP group, all with statistically significant differences (*P* < 0.05), as seen in Figure 1.

### 3.2. Comparison of Lung Function Parameters for Both Groups

Patients in the AE group had lower FEV1, FVC, FEV1/FVC, and FEV1% levels than those in the SP group, all with statistically significant differences (*P* < 0.05), as seen in Figure 2.

### 3.3. Correlation between *R* Value and Lung Function-Related Indicators in Patients with AECOPD

Correlation analysis showed that the *R* value in TEG of AECOPD patients was positively correlated with pulmonary function-related indicators (FEV1, FVC, FEV1/FVC, FEV1%) (*r* = 0.565, 0.529, 0.447, 0.527, all *P* < 0.001), as seen in Figure 3.

### 3.4. Correlation between *K* Value and Lung Function-Related Indicators in Patients with AECOPD

Correlation analysis showed that the *K* value in TEG of AECOPD patients was positively correlated with pulmonary function-related indicators (FEV1, FVC, FEV1/FVC, FEV1%) (*r* = 0.512, 0.567, 0.459, 0.439, all *P* < 0.001), as seen in Figure 4.

### 3.5. Correlation between *α*-Angle and Lung Function-Related Indicators in Patients with AECOPD

Correlation analysis showed that *α*-angle in TEG of AECOPD patients was inversely correlated with pulmonary function-related indicators (FEV1, FVC, FEV1/FVC, FEV1%) (*r* = −0.498, −0.372, −0.408, −0.424, all *P* < 0.001), as seen in Figure 5.

### 3.6. Correlation between MA Value and Lung Function-Related Indicators in Patients with AECOPD

Correlation analysis showed that MA value in TEG of AECOPD patients was inversely correlated with lung function-related indicators (FEV1, FVC, FEV1/FVC, FEV1%) (*r* −0.459, −0.429, −0.394, −0.403, all *P* < 0.001), as seen in Figure 6.

## 4. Discussion

Many studies [12–15] suggest that the body is in a long-term hypoxic state, which is easy to activate the coagulation system and promote the simultaneous occurrence of secondary fibrinolytic hyperfunction and hypercoagulability. Patients with AECOPD have long-term airflow restriction and hypoxia, resulting in an increase in the number of secondary red blood cells and a decrease in deformability, resulting in an increase in blood viscosity, promoting platelet adhesion and aggregation, and the formation of microthrombosis [16, 17]. There is no consensus on the indications for anticoagulation and the duration of anticoagulation in COPD patients. Therefore, the assessment of coagulation and fibrinolytic function in patients with AECOPD can provide an important reference for the anticoagulation treatment of COPD patients.

RETRACTED

TEG was invented by Hartert [18] of Germany in 1948 to image platelet aggregation through to thrombosis and subsequent fibrinolytic coagulation-fibrinolysis. Among them, the *R* value describes the content of coagulation factors in the blood, and the *K* value describes the speed of visible clot formation, which depends on thrombin, thrombin production, fibrinogen, and platelets; the *α*-angle indicates the rate of increase in clot strength over time and this variable correlates well with fibrinogen content; MA values reflect platelet function and clot-forming potency. In recent years, TEG has been widely used for coagulation-fibrinolytic function monitoring in clinical areas such as surgery, severe trauma, sepsis, and acute cerebral infarction [19–22].

In this study, patients with AECOPD and stable phase of COPD were tested for TEG and lung function and correlations were made between the relevant indicators, the results showed that the *R* and *K* values of patients in the AE group were lower than those in the SP group, and the *α*-angle and MA value were higher than those in the SP group, all with statistically significant differences (*P* < 0.05). This suggests increased coagulation factor activity, enhanced fibrinogen function, and enhanced platelet activity in patients with AECOPD. The *R* value reflects the coagulation factor activity and when it is lower than the normal reference value, it indicates enhanced coagulation factor activity [23]. Patients with COPD suffer from chronic hypoxia, inflammation, and CO_2_ retention, causing secondary erythropoiesis, increased erythrocyte pressure volume, and reduced erythrocyte deformability in the blood, resulting in slower blood flow, increased blood viscosity and concomitantly increased coagulation factor activity [24]. Spasms of pulmonary arterioles due to long-term hypoxia can cause pulmonary hypertension, poor systemic circulation, and blood stasis, which will further increase the activity of coagulation factors; At the same time, when the vascular endothelium of AECOPD patients is subjected to oxidative stress and inflammatory injury, the endothelial cell function is disordered, and the activated inflammatory cells release a large number of inflammatory mediators and inflammatory factors, which not only aggravate airway inflammation, but also activate the endogenous and exogenous coagulation system, increase the activity of coagulation factors, and make the patient's blood in a hypercoagulable state [25]. Both the *K* value and the *α*-angle reflect the fibrinogen function. When the *K* value is lower than the normal reference value or the alpha angle is higher than the normal reference value, it indicates enhanced fibrin activity or increased fibrinogen [26]. The enhanced fibrinogen activity in the patients enrolled in this study may be explained by the fact that during acute exacerbations of COPD, due to the presence of a hypercoagulable state of the blood, fibrinogen is not only involved in the endogenous and exogenous coagulation process as a coagulation factor but can also act as an acute phase response protein, triggering platelet aggregation and increasing blood viscosity; and elevated fibrinogen provides more substrates for enzymatic reactions in the coagulation process and also causes a marked increase in the aggregation of red blood cells, reducing the speed of blood flow and stagnation of blood, thus promoting thrombosis; In addition, recurrent lung infections and chronic inflammatory processes can also lead to increased fibrinogen and enhanced activity [27]. MA mainly reflects platelet function, and when MA is elevated it indicates increased platelet activity and a hypercoagulable state of blood [28]. Long-term hypoxia and inflammatory stimulation damage the vascular endothelial system of AECOPD patients, after endothelial damage, subintimal collagen fibers are exposed and release tissue factors, and platelets gather, which then affect the production of anticoagulant factors and the balance of the pulmonary vascular internal environment, so as to start endogenous and exogenous coagulation, resulting in the imbalance of coagulation function and fibrinolytic system; Inflammatory mediators and inflammatory factors released by inflammatory cells following damage to the vascular endothelium in patients with AECOPD, which not only damage lung tissue structure and increase airway inflammation but also interact with platelets and enhance platelet activity; In addition, chronic tobacco and toxic particle irritation can inhibit prostacyclin synthesis in the blood, which enhances the action of thromboxane A2, which can also trigger platelet aggregation and increase platelet activity [29].

RETRACTED

Pulmonary function tests are the main objective indicator of persistent airflow limitation and can reflect the severity of changes in COPD [30]. In this result, FEV1, FVC, FEV1/FVC, and FEV1% levels were lower in the AE group than in the SP group, and all differences were statistically significant (*P* < 0.05). This indicates a progressive decline in lung function as the COPD patient's condition worsens. Further analysis of the correlation between changes in TEG and pulmonary function-related indicators in AECOPD patients showed that the *R* and *K* values in TEG of AECOPD patients were positively correlated with pulmonary function-related indicators (FEV1, FVC, FEV1/FVC, FEV1%) (all *P* < 0.001), and the *α*-angle and MA value were inversely correlated with pulmonary function-related indicators (FEV1, FVC, FEV1/FVC, FEV1%) (all *P* < 0.001). This means that as the *R* and *K* values of AECOPD patients fall, the *α*-angle and MA value rise, their FEV1, FVC, FEV1/FVC, and FEV1% levels fall, airway resistance gradually increases, the more severe the lung tissue damage, and the condition continues to deteriorate.

## 5. Conclusion

TEG parameters can reflect the full range of dynamic changes in coagulation, and pulmonary function tests can be used to determine the severity of persistent airflow limitation. There is a correlation between TEG-related indicators and lung function-related indicators in AECOPD patients, both of which can guide the diagnosis and treatment process of the disease and are worthy of clinical promotion.

## Figures and Tables

**Figure 1:** Comparison of TEG parameters for both groups. Note: ^*∗*^ means the difference between groups for comparison, *P* < 0.05.

**Figure 2:** Comparison of lung function parameters for both groups. Note: ^*∗*^ means the difference between groups for comparison, *P* < 0.05.

**Figure 3:** Scatter plot of correlation between *R* value and FEV1, FVC, FEV1/FVC, and FEV1% in patients with AECOPD.

**Figure 4:** Scatter plot of correlation between *K* value and FEV1, FVC, FEV1/FVC, and FEV1% in patients with AECOPD.

**Figure 5:** Scatter plot of correlation between *α*-angle and FEV1, FVC, FEV1/FVC, and FEV1% in patients with AECOPD.

**Figure 6:** Scatter plot of correlation between MA value and FEV1, FVC, FEV1/FVC, and FEV1% in patients with AECOPD.

**Table 1:** Baseline information collection.

	AE group (*n* = 100)	SP group (*n* = 80)	*χ * ^2^ * /t* value	*P* value
Gender (*n*, %)			0.037	0.848
Male	75	59		
Female	25	21		
Smoking history (*n*, %)			0.001	0.972
Yes	64	51		
No	36	29		
Age ($\bar{x}$±*s*, years old)	63.41 ± 6.12	62.91 ± 6.51	0.529	0.597
BMI ($\bar{x}$±*s*, kg/m^2^)	22.75 ± 1.37	22.68 ± 1.41	0.336	0.737
Duration of illness ($\bar{x}$±*s*, years)	3.53 ± 1.05	3.62 ± 1.07	0.567	0.572
Days of exacerbation ($\bar{x}$±*s*, days)	4.29 ± 1.20	4.48 ± 1.22	1.048	0.296

**Table 2:** Reference ranges of TEG indicators and their significance for detection.

TEG indicator	Reference values	Significance for detection
*R* Value	5.00–10.00	Reflective of coagulation factor activity
*K* Value	1.00–3.00	Reflective of fibrinogen function
*α*-angle	53.00–72.00	Reflective of fibrinogen function
MA value	50.00–70.00	Reflective of platelet function

RETRACTED

## Data Availability

The data used or analyzed during the study are available from the corresponding authors upon reasonable request.
